The article "Prognostic Value of Stem Cell Index-Related Characteristics in Primary Hepatocellular Carcinoma" was retracted in 2023. Reasons: signs of a paper mill; suspected computer-generated content; unreliable results or conclusions; concerns about the data.

# Prognostic Value of Stem Cell Index-Related Characteristics in Primary Hepatocellular Carcinoma

**DOI:** 10.1155/2022/2672033

**Published:** 2022-06-08

**Authors:** Guihua Rao, Huifen Pan, Xia Sheng, Jin Liu

**Affiliations:** ^1^Department of Laboratory, Minhang Hospital, Fudan University, Shanghai 201199, China; ^2^Department of Pathology, Minhang Hospital, Fudan University, Shanghai 201199, China; ^3^Department of Gastroenterology, Minhang Hospital, Fudan University, Shanghai 201199, China

## Abstract

The objective of this study is to form a cancer stem cell index-based model to stratify HCC risk and predict survival. After screening the Tumor Genome Atlas (TCGA) of liver and normal liver tissue samples, we obtained differentially expressed genes (DEGs). We employed a weighted correlation network analysis (WGCNA) and differentially expressed genes were studied in HCC to find the modules most associated with cancer stem cells (mRNAsi). At the same time, gene ontology and Kyoto Genome Encyclopedia (KEGG) were used for functional annotation and combined with LASSO, univariate, and multivariate COX regression analyses, a prediction model of key module genes of cancer stem cells was developed. The model's clinical efficacy was measured using the C index, calibration curve, multiindex ROC curve, and clinical decision curve. WGCNA found that black modules were most correlated with tumour stem cell index. Seven genes (CSDC2, GNA14, LGI2, MMRN1, PDE2A, SELP, and STK32B) were filtered by univariate, LASSO, and multivariate Cox regression analyses to establish the primary HCC model. The survival analysis and ROC curve in the TCGA training and validation cohort showed good performance. The independent prognostic factor of primary HCC was risk score, according to univariate and multivariate Cox regression analyses. It is found that the stem cell index model of 7 genes could predict factors independently, indicating that signatures of the stem cell will play a significant role in liver cancer survival prediction and risk stratification.

## 1. Introduction

On deaths worldwide annually [1, 2], East and Southeast Asia and North and West Africa have a higher HCC incidence. China accounts for 50% of reported HCC cases [3–5]. Many main risk factors including hepatitis B or C infection, smoking, and aflatoxin exposure, contributed to hepatocellular carcinoma [6–9]. The main cause of hepatocellular carcinoma in non-alcoholic fatty liver disease (NAFLD) or obesity-related non-alcoholic steatohepatitis (NASH) is not clear, according to the findings of experts in recent years [10]. Through b-type ultrasound, serum alpha-fetoprotein (AFP) detection, and CT scan, currently, HCC could be diagnosed at an early stage, but it is often misdiagnosed [11]. Therefore, there is an urgent need to use a variety of molecular markers to identify and improve the prognosis of HCC.

The tumour cells with their self-renewal ability give rise to heterogeneous tumour cells known as cancer stem cells (CSC). In terms of tumour survival, propagation, transfer, and recurrence, cancer stem cells are of great importance. It is believed that fresh dryness indices were used to extract tumour dryness features, such as mRNA expression dryness index (mRNAsi) and DNA methylation dryness index [12]. There are few studies, however, that have tried to determine stem cell-related gene's prognostic and predictive significance in HCC. For assessing the mRNAsi score and using a kind of logistic regression machine learning algorithm, it is found that there is a serious correlation between mRNAsi and HCC prognosis. Under this circumstance, novel ideas are offered for studying stratified tumours with different clinical outcomes, which provides a new idea for the study of stratified tumours with diverse clinical findings [12]. Nevertheless, this concentrated on an all-around, wraparound cancer analysis. mRNAsi was significantly related to overall cancer survival, but the study was based only on general tumour levels. Other mRNAsi-related genes have not been specifically analysed, and their biological roles remind unclearly.

As a result, in HCC, differentially expressed genes (DEGs) were screened in this study from The TCGA database. Subsequently, we adopted the WGCNA to measure key gene clusters for the HCC stem cell index. Meanwhile, we annotated key modules of stem cells using the KEGG. Finally, a gene model associated with the HCC stem cell index was established, and the training set (60%) and internal validation set (40%) from the TCGA database were selected for validation.

## 2. Materials and Methods

### 2.1. Data Processing

We collected 424 HCC patients' high-throughput RNA-SEQ data by downloading them from the University of California, Santa Cruz (UCSC) Xena website. Based on fragment/graph read per million (FPKM) normalization estimates of fragments per thousand base pairs, we then quantified gene expression profiles by log2-based transformations. Furthermore, we applied the “Limma” software package in R software to screen differential genes. The screening criteria for differential genes in liver cancer were as follows: the absolute value of multiple changes (FC) of log2 conversion >1 and adjusted *P*-value (adj. *P*) <0.05.

### 2.2. mRNA-Seq Stem Cell Index Acquisition

Langfelder P, Maltese et al. [12] provided a novel analytical method to evaluate the carcinogenicity differentiation of HCC samples considering the mRNAsi. We used the first-order logistic regression machine learning algorithm (OCLR) of the TCGA HCC dataset to calculate the HCC samples' mRNAsi score, ranging from 0 (no gene expression) to 1 (complete gene expression). According to earlier studies, we got mRNAsi through multiplatform analysis.

### 2.3. WGCNA Constructs Stem Cell Index-Related Modules

For forming the gene co-expression similarity matrix and to develop gene co-expression networks, this study employed the WGCNA [13]. The absolute value of the Pearson correlation coefficient between gene *I* and gene *J* was first calculated, where *I* and *J* stand for gene *I* and gene *J* expression levels, respectively:

(1) $$\begin{array}{c} S_{ij}=\left|\frac{\left(1+\text{cor }\left(x_{i}+y_{j}\right)\right)}{2}\right|. \end{array}$$

Next, we converted the gene expression similarity matrix into an adjacency matrix for network type division. *β* is the Pearson correlation coefficient for each pair of genes and is the soft threshold:

(2) $$\begin{array}{c} a_{ij}={\left|\frac{\left(1+\text{cor }\left(x_{i}+y_{j}\right)\right)}{2}\right|}^{\beta }. \end{array}$$

Then we converted the adjacency matrix to a topological matrix. The degree of similarity between gene *I* and gene *J* is represented by TOM. 1-Tom is regarded as the distance for hierarchical genes clustering, and then used way of dynamically cutting trees for module identification:

(3) $$\begin{array}{c} \text{TOM}=\frac{\left(\sum_{\mu \neq ij}a_{iu}a_{uj}+a_{ij}\right)}{\left(\min\left(\sum_{\mu }a_{iu}+\sum_{\mu }a_{j\mu }\right)+1-a_{ij}\right)}. \end{array}$$

In each module, the feature vector gene (ME) refers to the most representative gene and represents the genes' overall expression level. *J* stands for microarray samples in module *Q*, and I stands for genes in module *Q*:

(4) $$\begin{array}{c} \text{ME}=\text{prin comp}\left(x_{ij}^{q}\right). \end{array}$$

We measured genes identity in modules by using the Pearson relation between the ME expression profiles of the intrinsic vector genes and the gene expression profiles of all samples. It is named module member (MM):

(5) $$\begin{array}{c} {\text{MM}}_{i}^{q}=\text{cor }\left(x_{i},{\text{ME}}^{q}\right). \end{array}$$

In the TCGA database, we initially used the HCC transcriptome as the data source. A prerequisite for the development of the WGCNA was a high-precision analysis of the correlation of the expression levels of 6962 DEGs. According to the correlation of each DEG, the parameter *β* was set, and a scale-free co-expression network was realized. Then, the “Blockwise” function is used for network construction and module detection. What is more, we studied the relationship between modules and mRNAsi scores, with modules identified by the most connected, highest ranked modules.

### 2.4. Gene Functional Enrichment Analysis

This study adopted the R software “cluster profile” package in the WGCNA analysis to take GO and KEGG enrichment analysis of genes in the most important modules [14].

### 2.5. Inclusion Criteria of HCC Patients with Stem Cell Index Risk Prognosis Model

The inclusion standard we adopted contained: (1) primary HCC patients (excluding recurrence); (2) whole clinicopathological features; (3) RNA sequencing data of samples can be obtained; (4) with OS as the essential endpoint; and (5) follow-up of at least 90 days. The exclusion standard was: (1) patients pathologically diagnosed with HCC recurrence; (2) patients with tumours other than HCC; and (3) absence of survival status and clinicopathological parameters.

### 2.6. Establishment of Stem Cell Exponential Prognostic Model

Univariate Cox regression analysis was conducted by R's “Survival” package to measure genes that are critical to survival and highly correlated with survival, and then further, we optimized the key prognostic genes by choosing the operator (LASSO) regression model and minimum absolute contraction [15]. Using R package, “GLMnet” was applied, and we found a boosted multivariate Cox regression analysis after key prognostic genes reduction and variable selection to produce risk score models. We built the formula based on the gene's coefficients and expression levels:

(6) $$\begin{array}{c} \text{Model}:\text{Risk score}=\sum \beta Si. \end{array}$$

*K* is the model gene number; Si is the key genes' expression level, and *β* is the coefficient index. After that, the software package “Survminer” was used to obtain the optimal critical value [16]. We randomly divided the patients with primary liver cancer in the TCGA dataset into a training group (60%) and an internal validation group (40%) by using the “CareT” package in the R software. We plotted time-dependent ROC curves using the Kaplan–Meier survival difference test to identify whether risk scores precisely predicted survival status. Lastly, the “Complex Heatmap” R program package was used to show the correlation between characteristic genes and individual HCC patients' risk scores in the Heatmap.

### 2.7. Prediction Ability of Internal Validation Set Analysis Model

We validated the external risk feature through the TCGG internal validation set data. We equally separated the samples into two groups with the same threshold and applied Kaplan–Meier analysis to assess both groups. The risk scores discriminability of the external validation set was then evaluated using ROC curve analysis. In addition, a risk heat map was then produced and presented the relationship between the distribution of prognostic model genes and the individual risk score of HCC patients.

### 2.8. Prognostic Value Evaluation of the Model

We used univariate and multivariate Cox regression analyses (covering histological grade, age, risk score, sex, pathological stage, and t-stage). We assessed whether the HCC patient prognostic model was independent of other clinicopathological variables. We set clinical characteristics as the independent variable, and calculated hazard ratios (HR), 95% confidence intervals, and *p*-values.

### 2.9. Expression Analysis of Model Genes

We adopted a two-sample *T*-test to analyse the distribution of gene expression in the model in the TCGA liver cancer microarray [17]. In addition, the publicly available human protein mapping (https://www.proteinatlas.org) to download the immunohistochemical image, is used to compare protein expression levels associated with the genetic model [18].

### 2.10. Establishment of Hepatocellular Carcinoma Survival Prediction Line Graph and Model Evaluation

An intricate statistical forecasting model was reduced to a rosette. We used it to assess the likelihood of OS in individual patients. One of the useful ways to forecast a cancer patient's prognosis is rosette [19]. From Cox regression analysis, we developed a graph that was able to evaluate the probability of 1-, 3-, and 5-year OS by choosing all independent clinicopathological prognostic factors. We checked the model's accuracy by measuring its effectiveness through multiindex ROC and clinical decision curves.

### 2.11. Statistical Analysis

We adopted R software (version 4.0.2) to carry out a statistical analysis of this experiment. For the selection of differentially expressed genes, we used the Wilcoxon test and Kaplan–Meier curve to study the distinction in survival between the two groups.

## 3. Results

### 3.1. Identification of Importance Modules of Stem Cell Index

As shown in Figure 1(a), mRNA expression profiles of normal tissues (*n* = 50) and the liver cancer tissues (*n* = 374) were compared and then analysed. Of the total 6961 differential genes, 5111 genes were upregulated and 1850 genes were downregulated. After data preprocessing, correlation analysis was performed on 6961 HCC differential genes with a soft threshold power of 6 for *β* to ensure a scale-free topological model, as shown in Figure 1(b). Then, we developed gene coexpression modules and appointed them into diverse modules using tree graphs, as shown in Figure 1(c).  Figure 1(d) shows the relationship coefficient between the stem cell index signature and each coexpressed gene module. By module and phenotypic correlation analysis, we found that the black module was most correlated with HCC stem cells (*R* = −0.70, *P* = 8*E* − 54). Therefore, the black module is considered to be the most important module that is most correlated with the stem cell index.

### 3.2. KEGG and GO Enrichment Analysis of Central Genes

Figure 2 shows the identification of functional gene annotation in the black module. The R software “cluster profile” package in the black modules was applied, and we conducted an enrichment analysis of genes. Based on KEGG pathway analysis, black module genes were primarily concentrated on ECM-receptor interaction, local adhesion, MAPK signalling pathway, Rap1 signalling pathway, hypertrophic cardiomyopathy (HCM), human papillomavirus infection, axon guidance, and cytogenesis Sub-the interaction of cytokines receptors, age-rage signalling pathway in diabetic complications, malaria, amoebiasis, dilated cardiomyopathy (DCM), phospholipase *D* in the signal transduction pathway, cancer protein, polysaccharide, arrhythmia, right ventricular cardiomyopathy (ARVC), and the interaction between neural activity ligand and receptor, TGF-beta signalling pathway, calcium signal transduction pathway, the regulation of actin cytoskeleton. GO analysis results show that the black module gene biological process mainly enriched in the extracellular matrix, the structure of the extracellular tissue, skeletal system development, participates in cell morphogenesis, the differentiation of neurons axon growth and development of the eyes, the growth of connective tissue, interstitial tissue of the development, development of the eyes, the visual system development, the development of the sensory system, ossification, axons organs, embryo development, chondrogenesis, glomerular vascular development, regulation of neuronal projection development, epithelial cell proliferation, embryonic organ morphogenesis, and cardiac morphogenesis.

### 3.3. Prognosis Model of Primary HCC

For genes in the black modules, univariate Cox regression analysis was conducted to figure out the prognostic value of genes along with stem cell index. We identified 60 genes greatly related to OS in primary liver cancer, as shown in Figure 3(a). We employed the “CareT” software package to divide primary liver cancer patients in the TCGA dataset into a training group (60%) and an internal validation group (40%) randomly to develop a clinical HCC survival and prognosis model. We first used the TCGA training set (60%) as the data set. We analysed 60 survival-related genes with LASSO Cox regression. We found that the most stable prognostic indicators were obtained by using relative regression coefficients. And cross-validation was performed to avoid overfitting with the LASSO Cox model, as shown in Figures 3(a) and 3(b). The parameters of the multivariate Cox model were established, and seven markers such as CSDC2, GNA14, LG12, MMRN1, PDE2A, SELP, and STK32 B were screened, as shown in Table 1. Then, according to the minimum criteria, we formed a polygenic model using seven genes. Subsequently, we used the coefficients obtained by the LASSO algorithm, comparing the survival status of the two groups of patients and the relationship of seven gene expressions, as shown in Figure 4(a). Next, we verified the predictive function of the seven genes in the internal validation set. Through the same formula in the validation set, a risk score was measured for each patient. The cutoff value was the median risk rating. The seven genes' survival and expression were compared between the two groups. Such outcomes also occurred in the training set: poorer outcomes were achieved in the high-risk group, as shown in Figure 4(b).

### 3.4. mRNA and Protein Expressions of Seven Genes in the HCC

In HCC, all six genes had an insufficient expression, compared with adjacent nontumour liver tissue in the TCGA HCC cohort. By analysing HCC clinical samples in the HPA database and the expression of the proteins that were encoded by the seven genes, we identified the clinical relevance of the expression of these seven genes. In contrast to normal liver tissues, CDSC2 was moderately expressed. But GNA14, LG12, MMRN1, PDE2A, and SELP were not expressed in HCC tissues, as shown in Figures 5(g)to 5(l). However, STK32B information is not available on the HPA website.

### 3.5. Survival Analysis and Time-Dependent ROC Curve Based on Seven-Gene Model

Two groups' overall survival (OS) is presented in the Kaplan–Meier survival curve. In addition, we applied the time-dependent area under the ROC curve (AUC) to evaluate the prognostic power of the seven-gene model, with a higher AUC indicating better model performance. In the TCGA training set (*P* < 0.0001), there was a remarkable distinction in OS between the two groups, as shown in Figure 6(a).The AUCs of the seven-gene models corresponding to the 1-, 3-, and 5-year survival rates are 0.76, 0.79, and 0.84, respectively.  Figure 6(c) presented a predictive model that has excellent sensitivity and specificity. Another Kaplan–Meier curve was presented compared to the lower risk group, and OS was a significantly higher internal validation set (*P* < 0.05), as shown in Figure 6(b). This finding was in line with our earlier outcomes from the training cohort.  Figure 6(d) presented that 0.65, 0.69, and 0.70 were the AUC scores corresponding to the 1, 3, and 5-year survival rates, respectively. The seven-gene model was further confirmed to have moderate sensitivity and specificity as a good OS predictor in HCC patients.

### 3.6. Prognostic Risk Score was an Independent Prognostic Factor for Other Clinicopathological Features

Univariate and multivariate Cox regression of HCC patients were shown in Figure 7, and the independent predictive significance was assessed and analysed. Univariate Cox regression indicated that in the TCGA training set, risk score, pathological stage, and *T*-stage existed prognostic significance, while there was no correlation between age, sex, histological grade, and survival, as shown in Figure 7(a). The only independent prognostic factor related to OS was risk score, as shown in Figure 7(c), according to multivariate Cox regression analysis. We further explored an independent prognostic marker for the HCC cohort in the TCGA internal validation set.  Figure 7(b) presented that there was a relationship between *t* stage, risk score, pathological stage, and OS.  Figure 7(d) suggested that existed a relationship between risk score and OS (*P* < 0.05). Independent predictors of prognosis in HCC patients could be according to the risk score of the seven-gene model, confirmed by these results.

### 3.7. Prognostic Value Evaluation of the Model

A graph was formed to forecast the probability of 1-, 3-, and 5-year OS in the TCGA cohort. Then, a clinically applicable predicting way for survival possibility in HCC patients was built. Six prognostic factors (age, sex, pathological stage, pathological grade, T-stage, and risk score) were used as predictors of the rosette, as shown in Figure 8(a). We confirmed Rosette's reliability by analysing the calibration curves and discovered that the predicted 1-, 3-, and 5-year survival rates of Rosette were closely related to the observed survival rates, as shown in Figure 8(b). Both C-index and multiindex ROC presented that clinical predictive performance was great in the model, as shown in Figures 8(c) and 8(d). The clinical decision curve shows that when the risk score is included alone, the net benefit for HCC patients is significantly improved, as shown in Figure 8(e) and Model2.

## 4. Discussion

Still, one of the most lethal malignancies globally is liver cancer because of its extremely complex molecular mechanisms. Because gene sequencing technology is constantly evolving, it has been found several underlying genetic indicators have predictive significance. There is an insufficient number of such markers. As a result, there is a requirement to screen out more and more precise biomarkers urgently to forecast liver cancer prognosis to promote the HCC prognosis. By studying one HCC cohort's gene expression profiles in TCGA, we determined differential genes between HCC samples and normal groups, and univariate, Lasso, and multivariate were used.

The analysis further narrowed the range of markers, and a model for calculating risk was established to predict the prognosis of HCC. What we found in our research is that there was a correlation between the high expression of MMRN, CSDC2, LG12, and STK32 B genes and the poor prognosis. There was a correlation between high expression of GNA14, PDE2A, and SELP and promoted prognosis. We adopted the model's ROC curve to assess the model's performance. According to the results, 0.76, 0.79, and 0.84 were the AUCs of the seven-gene model corresponding to 1-, 3-, and 5-year survival, respectively. It showed that the seven-gene model played a great role in the survival prediction performance. Then, independent prognostic factors that the seven-gene model outperformed traditional clinicopathological factors were not only demonstrated by us. Their ability to forecast survival in an external HCC cohort was also validated in the TCGA internal validation set.

Consequently, this study held the opinion that we could perform HCC recurrence based on a seven-gene risk scoring model. A rotograph is a tool for cancer disease assessment that probabilistic predictions can be realized by it. We formed a garland that could forecast HCC patients' OS. According to the modified curve, there was a substantial agreement between the actual survival rate observed in the data and the set survival rate predicted by the line graph, suggesting that there was an excellent performance in the line graph. Meanwhile, the rosette had great predictive performance, according to the multiindicator ROC, clinical decision curve, and C-index.

HCC occurs through several pathway activation and molecular modifications, and it is a heterogeneous tumour. Meanwhile, lots of reports have discovered that there was a correlation between the low survival rate and the cells' stable propagation and anti-apoptotic gene expression, and diverse genes were always included in these processes. Polygenic markers existed with higher predictive power for HCC than single-gene markers [20]. Predicting the prognosis of HCC is usually performed by bioinformatics methods, which are often used to build polygenic models. Polygenic models are usually established through training sets and validation strategies within sets [21]. These strategies can significantly improve the predictive ability of gene models. It has been reported that the polygenic model has an excellent prediction impact on the venous metastasis, progression, recurrence, and survival of HCC [22–25]. According to the new seven-gene model, a higher 5-year survival prediction AUC (0.84) was developed in this study. There are few reports of a survival prediction model according to this seven-gene model. The polygenic model has more personalized detection outcomes, higher prediction accuracy, and reasonable sequencing cost than traditional pathological staging and tissue grading. As a result, in clinical practice, there are promising prospects for the seven-gene model. Our findings are more reliable if more rational use of biometric methods is used, and multiple independent datasets are mutually validated.

This study, however, has certain insufficiencies. The model was supposed to exclude ethnicity and some potential prognostic factors related to the sequenced samples, which imposed certain limitations on the model's predictive power. We hope that more sophisticated bioinformatics strategies can be used to improve the model in the future.

In conclusion, the findings presented for predicting OS, a great tool in HCC patients is a seven-gene-based prognostic model, and the lithograph containing the seven-gene model could be beneficial in clinical practice for the development of personalized HCC therapy.

## Figures and Tables

**Figure 1:** (a) Volcanic map showing differentially expressed genes in hepatocellular carcinoma samples, (b) WGCNA soft threshold selection, (c) clustering tree of genome-wide genes in hepatocellular carcinoma samples, and (d) relationship between modules and stem cell index phenotypes.

**Figure 2:** Identification of functional gene annotations in the black module (a) KEGG pathway enrichment analysis; (b) gene ontology—biological process analysis.

**Figure 3:** (a, b) The process of establishing A model containing the seven genes most associated with overall survival (OS) in the training set. Hazard ratios (HRs) and 95% confidence intervals (CIs) calculated by univariate Cox regression and coefficients calculated by multivariate Cox regression using LASSO are shown.

**Figure 4:** (a) Risk score distribution, survival overview, and gene expression heat map for (b) Risk score distribution, survival overview, and gene expression heat map for patients in the TCGA internal validation concentration.

**Figure 5:** (a)–(g) mRNA expression levels of seven-gene markers (conducted in TCGA database). (h)–(m) Human protein profile CSDC2, GNA14, LG12, MMRN1, PDE2A, and SELP in normal and hepatocellular carcinoma tissues ^*∗*^*P* < 0.05^*∗∗*^*P* < 0.01.

**Figure 6:** Based on risk scores (a, b), Kaplan–Meier overall survival (OS) curves of patients were divided into two groups in the TCGA training set and TCGA internal validation set. In the training and validation cohorts, there is a poorer OS in high-risk score patients (c, d). According to the ROC curve, the patient risk scores' predictive efficiency on the TCGA training set and the TCGA internal validation set for survival are shown.

**Figure 7:** (a)–(d) Univariate/multivariate Cox regression analysis of the correlation between clinicopathological factors (including risk score) and overall survival (OS) in TCGA patients.

**Figure 8:** (a) A calibration plot of A (b)–(d) rosette combining risk score and clinicopathological features, A C-index, multiindicator ROC, and clinical decision curve showing the predictive performance of the model.

**Table 1:** Genetic parameters in multivariate COX model.

Gene	Coef	HR	HR.95L	HR.95H	*p*-value
CSDC2	0.149	1.161	1.000	1.347	0.048
GNA14	−0.292	0.746	0.598	0.930	0.009
LGI2	0.177	1.194	1.004	1.420	0.044
MMRN1	0.269	1.309	1.090	1.571	0.003
PDE2A	−0.228	0.795	0.623	1.016	0.066
SELP	−0.229	0.794	0.676	0.934	0.005
STK32B	0.310	1.363	1.134	1.638	0.0009

## Data Availability

The simulation experiment data used to support the findings of this study are available from the corresponding author upon request.

## References

[1] Zhang Q., He Y., Luo N. (2019). Landscape and dynamics of single immune cells in hepatocellular carcinoma. *Cell*.

[2] El-Serag H. B., Rudolph K. L. (2007). Hepatocellular carcinoma: epidemiology and molecular carcinogenesis. *Gastroenterology*.

[3] Stockdale A. J., Chaponda M., Beloukas A. (2017). Prevalence of hepatitis D virus infection in sub-Saharan Africa: a systematic review and meta-analysis. *Lancet Global Health*.

[4] Apata I. W., Averhoff F., Pitman J. (2014). Progress toward prevention of transfusion-transmitted hepatitis B and hepatitis C infection--sub-Saharan Africa, 2000-2011. *MMWR Morb Mortal Wkly Rep*.

[5] Bosetti C., Turati F., La Vecchia C. (2014). Hepatocellular carcinoma epidemiology. *Best Practice & Research Clinical Gastroenterology*.

[6] Fan J. H., Wang J. B., Jiang Y. (2013). Attributable causes of liver cancer mortality and incidence in China. *Asian Pacific Journal of Cancer Prevention*.

[7] de Martel C., Maucort-Boulch D., Plummer M., Franceschi S. (2015). World wide relative contribution of hepatitis B and C viruses in hepatocellular carcinoma. *Hepatology*.

[8] Schaper M., Rodriguez-Frias F., Jardi R. (2010). Quantitative longitudinal evaluations of hepatitis delta virus RNA and hepatitis B virus DNA shows a dynamic, complex replicative profile in chronic hepatitis B and D. *Journal of Hepatology*.

[9] Petrick J. L., Braunlin M., Laversanne M., Valery P. C., Bray F., McGlynn K. A. (2016). International trends in liver cancer incidence, overall and by histologic subtype, 1978-2007. *International Journal of Cancer*.

[10] Thein H. H., Qiao Y., Zaheen A. (2017). Cost-effectiveness analysis of treatment with non-curative or palliative intent for hepatocellular carcinoma in the real-world setting. *PLoS One*.

[11] Malta T. M., Sokolov A., Gentles A. J. (2018). Machine learning identifies stemness features associated with oncogenic dedifferentiation. *Cell*.

[12] Langfelder P., Horvath S. (2008). WGCNA: an R package for weighted correlation network analysis. *BMC Bioinformatics*.

[13] Yu G., Wang L. G., Han Y., He Q. Y. (2012). clusterProfiler: an R Package for comparing biological themes among gene clusters. *OMICS: A Journal of Integrative Biology*.

[14] Tibshirani R. (1997). The lasso method for variable selection in the Cox model. *Statistics in Medicine*.

[15] Li M., Spakowicz D., Burkart J. (2019). Change in neutrophil to lymphocyte ratio during immunotherapy treatment is a non-linear predictor of patient outcomes in advanced cancers. *Journal of Cancer Research and Clinical Oncology*.

[16] Blum A., Wang P., Zenklusen J. C. (2018). SnapShot: TCGA-analyzed tumors. *Cell*.

[17] Uhlen M., Oksvold P., Fagerberg L. (2010). Towards a knowledge-based human protein Atlas. *Nature Biotechnology*.

[18] Park S. Y. (2018). Nomogram: an analogue tool to deliver digital knowledge. *The Journal of Thoracic and Cardiovascular Surgery*.

[19] Lee J. S., Chu I. S., Heo J. (2004). Classification and prediction of survival in hepatocellular carcinoma by gene expression profiling. *Hepatology*.

[20] Roessler S., Jia H. L., Budhu A. (2010). A unique metastasis gene signature enables prediction of tumor relapse in early-stage hepatocellular carcinoma patients. *Cancer Research*.

[21] Budhu A., Jia H. L., Forgues M. (2008). Identification of metastasis-related microRNAs in hepatocellular carcinoma. *Hepatology*.

[22] Kurokawa Y., Matoba R., Takemasa I. (2004). Molecular-based prediction of early recurrence in hepatocellular carcinoma. *Journal of Hepatology*.

[23] Hoshida Y., Villanueva A., Sangiovanni A. (2013). Prognostic gene expression signature for patients with hepatitis C–related early-stage cirrhosis. *Gastroenterology*.

[24] Li W., Lu J., Ma Z., Zhao J., Liu J. (2020). An integrated model based on a six-gene signature predicts overall survival in patients with hepatocellular carcinoma. *Frontiers in Genetics*.

[25] Zhang M., Wang X., Chen X., Guo F., Hong J. (2020). Prognostic value of a stemness index-associated signature in primary lower-grade glioma. *Frontiers in Genetics*.

